# Observation on the Efficacy of Shouhui Tongbian Capsule in the Treatment of Functional Constipation and Study on Its Regulatory Effect on Intestinal Flora

This article has been retracted.

**DOI:** 10.1155/2021/9024919

**Published:** 2021-11-01

**Authors:** Hongxi Zhang, Bao Han, Zhiyun Zhang, Zhenguo Tian, Yongduo Yu

**Affiliations:** ^1^Department of Anorectal, The Third Affiliated Hospital of Liaoning University of Traditional Chinese Medicine, Shenyang 110005, Liaoning, China; ^2^Department of Anorectal Surgery, Beijing Mayinglong Changqing Anorectal Hospital, Beijing 100195, China; ^3^Anorectal Department, Kunming Municipal Hospital of Traditional Chinese Medicine, Kunming 650011, Yunnan, China

## Abstract

Functional constipation is relatively common in both adults and children, exhibiting similar symptoms. However, there are significant differences in the epidemiology, symptomatology, pathophysiology, diagnostic tests, and treatment management of functional constipation by age. The treatment of functional constipation is generally based on lifestyle interventions, pelvic floor interventions, and pharmacotherapy. Pharmacological treatment is popular as the most direct and effective modality, especially the herbal preparations (e.g., Shouhui Tongbian capsule), which are popular for their lower toxic side effects and less physiological reactions. In our clinical study, patients with functional constipation who took Shouhui Tongbian capsules for a longer period of time showed significantly better improvement than those who took them for a shorter period of time (*P* < 0.001). Relative to the duration of the disease, the improvement effect was higher in patients with short duration of the disease than in patients with long duration of the disease (*P* < 0.001). What's more, Shouhui Tongbian capsule had a regulating effect on intestinal flora, and the regulating effect was stronger in patients with a shorter disease duration.

## 1. Introduction

Chronic constipation is a common disease caused by many reasons. Among them, constipation caused by abnormal function of the large intestine and anus is called functional constipation [1–3]. It is clinically regarded as an independent disease, which is characterized by decreased frequency of defecation, difficulty in defecation, incomplete defecation, dry and hard stool, and presence of no organic disease by barium enema or colonoscopy [4–6]. At present, the prevalence of functional constipation is about 2%–27% [7]. Constipation not only causes common anal diseases such as anal fissure and hemorrhoids, but also causes the occurrence and development of cardiovascular and cerebrovascular diseases. In severe cases, it can also cause colon cancer, which is life-threatening [8–10].

Functional constipation can be divided into slow transit constipation (STC), outlet obstructive constipation (OOC), and mixed constipation (MC) according to the characteristics of colon dynamics and the location of its occurrence [11]. STC is constipation caused by colonic dyskinesia that slows down the discharge of the contents in the intestine or stays in the colon [12]. OOC is an anorectal dysfunction caused by nonorganic factors, but its intestinal dynamics and function are normal [13]. However, the cause and mechanism of functional constipation in modern medicine have not yet been clarified [14]. So far, there has been no effective, long-term, and low side-effect medicine for the treatment of functional constipation. In general, patients with functional constipation are usually treated with laxatives [15–17]. However, long-term use of laxatives will cause patients to develop drug resistance and cause serious intestinal diseases, such as “laxative colon” and “colon melanosis”. As a result, the patient's condition deteriorates, simple constipation becomes complicated, and the recovery will be longer and difficult. In addition, when the drug treatment is not ideal, surgical treatment is also needed, which affects the patient's body function [18].

Among the causes of constipation, the intestinal flora occupies an important position. There are thousands of microorganisms in the intestinal tract of normal people, which are combined into intestinal flora according to certain rules, which restrict and interdepend on each other and build a biological barrier to prevent pathogenic bacteria from entering the body and maintain the health of the body [19]. Once the intestinal flora is out of balance, it will cause a variety of diseases and accelerate the body's aging. In addition, due to the different causes of constipation, the changes in the intestinal flora are also different. Compared with normal people, patients with constipation usually have more potentially lethal bacteria and decreased obligate anaerobic bacteria in their intestinal flora [20].

Chinese medicine has a unique theoretical basis for the study of constipation, as well as thousands of years of clinical treatment experience in which Chinese herbs such as atractylodes macrocephala, radix polygoni, aloe vera, and fructus lycii have exhibited certain therapeutic effects on constipation. The prescription of Shou Hao laxative capsules is composed of herbal ingredients such as atractylodes macrocephalae, agaricus, He Shou Wu, semen cassia, ginseng, aloe vera, wolfberry, and bitter orange. Clinical practice has proved that the drug has a fast curative effect, definite curative effect, no toxic side effects, especially for functional constipation. At the same time, in order to verify its safety, effectiveness, and regulation of intestinal flora in clinical treatment, we conducted a multicenter, prospective, and noninterventional real-world study from May 2018 to June 2019 clinical trials.

## 2. Materials and Methods

### 2.1. General Data Analysis

This is a multicenter, prospective, and nonintrusive real-world study conducted in 30 centers to observe the efficacy of Shouhui laxative capsules in treating 2396 patients with dysfunctional convulsion for 14 successive days over a period of 4 months. The programme was given clearance by the appropriate ethical board. Prior to treatment, all the participants were provided with information regarding the study in detail, and they voluntarily signed the well-informed consent form.

### 2.2. Inclusion and Exclusion Criteria

Inclusion criteria are as follows: the patients should be 18−80 years old, should meet the Rome III diagnostic criteria for functional constipation [21], should meet the diagnostic criteria for deficiency of both qi and yin and toxins in traditional Chinese medicine treatment, and should take the Shouhui Tongbian capsule for at least one course of treatment. All patients participated in the study voluntarily.

The exclusion criteria are as follows: the cause of functional constipation is caused by organic disease; patients with secondary constipation with a clear cause; women who are pregnant or breastfeeding; patients who have used functional constipation drugs in the past two weeks; patients with abnormal liver function with ALT, AST > 3ULN; or the patient is allergic or allergic to the treatment drug.

### 2.3. Treatment Method

This is a noninterventional study and, therefore, before deciding to include subjects in the study, the subjects should be given Hao laxative capsules (Lunan Hou Pu Pharmaceutical Co. Ltd.) separately for treatment in accordance with the relevant hospital regulations and ensure that all procedures performed at these visits are in accordance with usual clinical practice. Patients are given seven days of therapeutic medication at each visit, while the drug manager is required to complete the clinical trial dosing record form on time. The addition of other Western and Chinese medicines with similar efficacy to the drug under test is prohibited during the trial. The mechanism of action of the drug on functional constipation is also shown in Figure 1.

### 2.4. Evaluation Index

#### 2.4.1. Effectiveness Evaluation

Intestinal function Wexner score is the main indicator used to evaluate the therapeutic effect of Shouhui Tongbian capsule on functional constipation. According to the number of bowel movements, completeness (incomplete evaluation of sensation), degree of difficulty in defecation (assessment of pain), abdominal pain, time of going to the toilet, form of assistance, and cumulative number of defecation failures within 24 h, 0–30 points will be given, respectively. *Rating*. The lower the score, the milder the condition, and correspondingly, the higher the score, the more severe the condition. The observation indexes are observed and recorded before the experiment and the 8th day and the 15th day after the experiment.

The secondary treatment index is the quality of life scale for patients with constipation (PAC-QOL). PAC-QOL has been developed into a Chinese version with a total of 28 items, which involves patients' physiology, anxiety, social psychology, and satisfaction. The five-point Likert method is used for alternative answers. The degree is divided into five levels: none, mild, normal, severe, and very severe. The same is true for frequency, for example, none, occasionally, sometimes, often, and always. It corresponds to the 5 levels from 0 to 5 points. At the same time, the long-term effects of the Shouhui Tongbian capsule on patients with functional constipation of different courses are observed.

#### 2.4.2. The Occurrence of Adverse Events and Adverse Reactions

During treatment, it is necessary to closely observe the occurrence of adverse reactions of patients in each course, and accurately record the time of occurrence, the degree of occurrence of adverse reactions, the treatment process, and treatment results of adverse reactions that have occurred, and pay attention to whether there are serious adverse events. According to the 5-level criteria of affirmative, possible, possible, possibly irrelevant, and irrelevant provided by the Adverse Drug Reaction Monitoring Center of the Ministry of Health, the causal relationship between adverse events and experimental drugs was evaluated.

#### 2.4.3. Intestinal Flora Detection

The patient's feces were collected before and after the treatment and placed on a glass slide to push it flat. After it is naturally dried, it is fixed with flame, stained with gram, and observed under a microscope. The ratios of Gram-positive and negative bacilli, Gram-positive and negative cocci, and bacilli/coccus in the stool of patients before and after treatment were recorded.

### 2.5. Statistical Analysis

Statistical analysis was performed using SPSS 19.0. The student' t test was used to compare the differences in related indicators and TCM syndrome scores of the subjects before and after the intervention of the Shouhui Tongbian capsule. The Chi-square test is used for data statistics. *P* < 0.05 is statistically significant.

## 3. Results and Discussion

### 3.1. General Data Analysis

A total of 2396 cases were included, of which 47% were males and 53% were females. The average age was 50.6 ± 14.9 years, the average height was 166.1 ± 7.3 cm, the average weight was 64.0 ± 11.3 kg, the average body mass index was 23.1 ± 3.3 kg/m^2^, and the average course of disease was 465.6 ± 104.3 months. Among them, 0–6 months and 1–5 years had the largest number of patients, accounting for 32.4% and 37.4% of the total number, respectively. Patients with 7 to 12 months and more than 5 years accounted for 15.9% and 14.3%, respectively. Before admission, Wexner's average score was 12.4 ± 4.8. 23.7% of patients had received Western medicine treatment, and only 16.5% of patients had received TCM treatment (Figure 2).

### 3.2. Analysis of TCM Syndromes of Patients with Different Constipation Durations

According to the duration of constipation, patients were divided into four groups. It can be seen from Table 1 that most patients have bowel movements twice a week with the highest proportion of patients having a disease course of more than 5 years (*P* < 0.001). The longer the course of the disease, the lower the rate of 1–2 bowel movements every 1–2 day. Most patients have difficulty defecation sometimes or often. Among them, the longer the course of the disease, the higher the proportion of patients who often have difficulty in defecation (*P* < 0.001). Most patients spend 10–20 minutes on the toilet, and the proportion of patients who spend more than 30 minutes on the toilet increases with the length of the disease (*P* < 0.001). In addition, with the continuous increase in the course of the disease, the proportion of patients who need assisted defecation also gradually increased (*P* < 0.001). Only 24.4% of patients with a course of 0–6 months needed stimulant laxatives, and 44.7% of patients with a course of more than 5 years needed stimulant laxatives.

### 3.3. Wexner Score of Patients with Different Durations of Constipation

The Wexner scores of the four groups are shown in Figure 3. The comparison between groups showed that the longer the course of functional constipation, the higher the Wexner score. The Wexner score was highest in patients with a disease course of more than 5 years (*P* < 0.001). Comparing the results within the group, we can find that there is a negative correlation between the medication time and the Wexner score. The longer the time, the lower the Wexner score. After 14 days of treatment, the Wexner scores of each group were significantly lower than before and 7 days after treatment (*P* < 0.001). Patients with a disease course of more than 5 years have the lowest clinical recovery rate (only 27.5%), but nearly 49.4% of patients have significantly improved their symptoms, accounting for the highest proportion.

### 3.4. TCM Syndrome Curative Effect Score

Figure 4 shows the efficacy scores of the four groups of TCM symptoms. The comparison between groups showed that within 7 days of treatment, patients with a disease course of 1 to 5 years had the highest scores (*P* < 0.001). On the 14th day of medication, patients with a course of more than 5 years had the highest scores on the efficacy of TCM symptoms. In addition, the results within the group were compared. With the increase in medication time, the score of the TCM syndrome curative effect showed a declining trend (*P* < 0.001). Patients with a course of more than 5 years had the lowest clinical recovery rate (29.1%) and the highest rate of symptom improvement (34.2%).

### 3.5. Quality of Life of Patients with Different Durations of Constipation

The PAC-QOL of the four groups are shown in Figure 5. The results of the comparison between groups showed that the scores of patients with a course of 1 to 5 years before treatment were higher than those of other groups (*P* < 0.001). At the end of the second, eighth, tenth, and twelfth treatment, patients with a course of more than 5 years had the highest quality of life scores (*P* < 0.05). After comparing the results of PAC-QOL in patients with different course of disease, it was found that the scores of patients with 1 ∼ 5 years of course of disease before treatment were higher than those in other groups (P < 0.001).

### 3.6. Patient Satisfaction Scores for Different Durations of Constipation

The satisfaction scores of the four groups of patients are shown in Figure 6. The results of comparison between groups showed that patient satisfaction increased with the course of the disease, and patients with a course of more than 5 years had the highest satisfaction (*P* < 0.001). The results of the comparison within the group proved that with the extension of treatment time, patient satisfaction decreased (*P* < 0.001).

### 3.7. Safety Evaluation

The results of the safety evaluation are shown in Figure 7. 81.2% of the patients considered the safety level of this study to be level 1, and 99% of the patients had no adverse events. Therefore, the Shouhui Tongbian capsule in this study had no adverse effects on safety.

### 3.8. Changes in Intestinal Flora

In order to assess the changes in the intestinal flora of each group of patients before and after treatment, the proportions of each bacterial species were recorded (Figure 8). The results showed that the proportions of Gram-positive bacilli and bacilli/cocci increased in each group of patients after treatment, and the proportions of Gram-positive cocci, Gram-negative bacilli, and Gram-negative cocci decreased. This proves that the Shouhui Tongbian capsule can effectively improve the intestinal flora imbalance caused by functional constipation. In addition, comparing the results of the four groups, it can be found that the Shouhui Tongbian capsule is more effective in treating patients with a shorter course of disease.

### 3.9. Discussion

Due to the accelerating pace of modern life, increasing work pressure, and huge changes in eating habits, more and more people are prone to chronic constipation. At present, the cause of functional constipation is not fully understood. However, enteric neuropathy, smooth muscle degeneration, central neuropathy, and gastrointestinal hormone abnormalities are related to the etiology [22].

Chinese medicine believes that the most direct cause of constipation is the virtual-based large intestine conduction dysfunction and excess [23]. The pathogenesis of patients with large intestinal hyperconductivity is mostly gastrointestinal stasis, which can be divided into gastrointestinal heat, air stagnation, and cold stagnation. The etiopathogenesis of the patient with deficient conduction capacity of the large intestine is mostly associated with dryness of the bowels and poor movements, mainly consisting of Yin and Yang deficiencies and Qi and blood deficiencies. Even though there are many contributing factors to the functional constituency, the main clinical presentation is deficiency-heat. Therapy is typically a combination of weakness and reality.

The Shouhui Tongbian capsule used in this study is composed of Atractylodes macrocephala, donkey-hide gelatin, polygonum multiflorum, cassia, ginseng, aloe, wolfberry, and bitter orange. The results of modern pharmacological studies on the main ingredients show that, as the main active ingredients in polygonum multiflorum, anthraquinone compounds can effectively enhance intestinal peristalsis and have obvious laxative effects [24]. Aloin, an effective ingredient in aloe vera, can be converted into aloe-emodin, which can promote intestinal peristalsis through hydrolysis [25]. The results of studies on the pharmacological effects of Cassia seed show that it can last and moderately improve the problems of hypertension and hyperlipidemia in patients, and at the same time have a laxative effect [26].

Ejiao has the effects of nourishing blood, nourishing yin, and moisturizing dryness [27]. Lycium barbarum has a nourishing effect on liver, lungs, and kidneys in Chinese medicine research. It is a good medicine for the treatment of intestinal dryness and constipation [28]. In addition to promoting gastrointestinal secretion and increasing peristaltic action, atractylodes macrocephala can also effectively regulate the already disordered intestinal flora [29]. In addition to stimulating peristaltic movement, agaric oranges have a relaxing effect on the smooth muscles of the intestine.

The advantage of the Shouhui Tongbian capsule is that it combines polygonum multiflorum with aloe vera, which enhances the functions of clearing away heat, detoxifying, and moisturizing the intestines. Dietary fiber and Western medicine are usually used to treat constipation. However, it has been reported that increasing the intestinal water content cannot shorten colonic transit time, and dietary fiber may cause bloating and hardened stools [30]. Western medicine treatment of constipation has disadvantages such as large side effects and poor tolerance, and there is no progress at present. Therefore, the treatment of constipation with traditional Chinese medicine has become a research hotspot at this stage.

This study compared the therapeutic effects of the Shouhui Tongbian capsule on patients with functional constipation of different courses through actual research on a large sample. The results of the study prove that the Shouhui Tongbian capsule can significantly improve the number of defecations, the nature of defecation, and the degree of difficulty in defecation, and the improvement effect gradually increases with the extension of the treatment time. However, the defecation effect of patients with a shorter course is better than those with a longer course (*P* < 0.001). The results of life, quantity, and patient satisfaction showed that prolonging the duration of medication significantly improved the life quality and contentment of patients. In addition, it has a more obvious improvement effect on patients with a shorter course of disease (*P* < 0.01). In addition, by detecting the changes in the intestinal flora of patients with different disease courses and time, it can be found that patients with a shorter course of disease have a more obvious regulatory effect on the intestinal flora. In summary, the findings of this study provide a new basis for choosing the time and frequency of medication for patients with functional constipation in different courses.

## 4. Conclusion

This study investigated the therapeutic effects of Shouhui Tongbian capsules on patients with functional constipation in different courses of treatment through various indicators such as effectiveness, quality of life of patients, and intestinal flora regulation ability. Functional constipation has a significant improvement effect, and the effect is better for patients who have a shorter treatment course and regulated intestinal flora. No obvious side effects and adverse reactions have been seen in clinical trials. It provides a new basis for choosing the timing and frequency of medication for patients with functional constipation of different courses and lays a foundation for the follow-up mechanism research [31].

## Figures and Tables

**Figure 1:** The mechanism diagram of the Shouhui Tongbian capsule on functional constipation.

**Figure 2:** Demographic characteristics of subjects.

**Figure 3:** Effect of Shouhui Tongbian capsule on Wexner's constipation score in patients with different courses (^*∗*^*P* < 0.001). (a) Wexner constipation score of patients. (b) Evaluation of the curative effect of Shouhui Tongbian capsule on patients with different courses.

**Figure 4:** The effect of Shouhui Tongbian capsule on the treatment effect of TCM symptoms in patients with different courses of treatment (^*∗*^*P* < 0.001). (a) TCM symptom therapeutic effect score in patients. (b) Evaluation of the treatment effect of the Shouhui Tongbian capsule in traditional Chinese medicine.

**Figure 5:** Patient quality of life score.

**Figure 6:** Patient satisfaction evaluation.

**Figure 7:** Patient safety evaluation. (a) Patient safety rating evaluation. (b) The occurrence of adverse reactions in patients.

**Figure 8:** The regulating effect of the Shouhui Tongbian capsule on the intestinal flora of patients with different courses. (a) 0–6 months. (b) 6–12 months. (c) 1–5 years. (d) >5 years.

**Table 1:** TCM symptoms for different durations of constipation.

	0–6 months (*N* = 776)	7–12 months (*N* = 381)	1–5 years (*N* = 897)	More than 5 years (*N* = 342)	*P* value
Frequency of defecation *n* (%)					
1–2 times per 1–2 days	194 (25.0%)	68 (17.8%)	103 (11.5%)	43 (12.6%)	< 0.001
Twice a week	310 (39.9%)	160 (42.0%)	376 (41.9%)	157 (45.9%)	
Once a week	164 (21.1%)	91 (23.9%)	265 (29.5%)	94 (27.5%)	
Less than once a week	106 (13.7%)	59 (15.5%)	147 (16.4%)	46 (13.5%)	
Less than once a month	2 (0.3%)	3 (0.8%)	6 (0.7%)	2 (0.6%)	

Difficulty: pain assessment *n* (%)					
Never	81 (10.4%)	36 (9.4%)	47 (5.2%)	36 (10.5%)	< 0.001
Very seldom	216 (27.8%)	93 (24.4%)	186 (20.7%)	64 (18.7%)	
Sometimes	262 (33.8%)	138 (36.2%)	316 (35.2%)	121 (35.4%)	
Often	169 (21.8%)	84 (22.0%)	280 (31.2%)	94 (27.5%)	
Always	48 (6.2%)	30 (7.9%)	68 (7.6%)	27 (7.9%)	

Integrity: incomplete sensory assessment, *n* (%)					
Never	73 (9.4%)	30 (7.9%)	47 (5.2%)	21 (6.1%)	< 0.001
Very seldom	221 (28.5%)	76 (19.9%)	170 (19.0%)	49 (14.3%)	
Sometimes	240 (30.9%)	148 (38.8%)	290 (32.3%)	133 (38.9%)	
Often	192 (24.7%)	97 (25.5%)	321 (35.8%)	104 (30.4%)	
Always	50 (6.4%)	30 (7.9%)	69 (7.7%)	35 (10.2%)	

Pain: abdominal pain *n* (%)					
Never	109 (14.0%)	59 (15.5%)	96 (10.7%)	52 (15.2%)	0.0845
Very seldom	254 (32.7%)	121 (31.8%)	240 (26.8%)	103 (30.1%)	
Sometimes	268 (34.5%)	131 (34.4%)	331 (36.9%)	119 (34.8%)	
Often	118 (15.2%)	53 (13.9%)	201 (22.4%)	53 (15.5%)	
Always	27 (3.5%)	17 (4.5%)	29 (3.2%)	15 (4.4%)	

Time: time on the toilet (minutes) *n* (%)					
Less than 5	34 (4.4%)	9 (2.4%)	11 (1.2%)	7 (2.0%)	< 0.001
5–10	184 (23.7%)	82 (21.5%)	181 (20.2%)	61 (17.8%)	
10–20	308 (39.7%)	177 (46.5%)	374 (41.7%)	144 (42.1%)	
20–30	176 (22.7%)	81 (21.3%)	234 (26.1%)	88 (25.7%)	
More than 30	74 (9.5%)	32 (8.4%)	97 (10.8%)	42 (12.3%)	

Auxiliary: auxiliary form *n* (%)					
No	486 (62.6)	238 (62.5%)	455 (50.7%)	113 (33.0%)	< 0.001
Irritant laxatives	189 (24.4%)	103 (27.0%)	300 (33.4%)	153 (44.7%)	
Finger assistance or enema	101 (13.0%)	40 (10.5%)	142 (15.8%)	76 (22.2%)	

Failure: number of failed attempts to defecate 24 hours *n* (%)					
No	130 (16.8%)	74 (19.4%)	121 (13.5%)	45 (13.2%)	0.001
1–3 times	418 (53.9%)	219 (57.5%)	497 (55.4%)	189 (55.3%)	
3–6 times	161 (20.7%)	56 (14.7%)	228 (25.4%)	84 (24.6%)	
6–9 times	58 (7.5%)	27 (7.1%)	39 (4.3%)	16 (4.7%)	
More than 9 times	9 (1.2%)	5 (1.3%)	12 (1.3%)	8 (2.3%)	

## Data Availability

The data underlying the results presented in the study are available within the article.
